The article "Design and Analysis of Clothing Catwalks Taking into Account Unity's Immersive Virtual Reality in an Artificial Intelligence Environment" was published in 2022. Journal: Comput Intell Neurosci.

# Design and Analysis of Clothing Catwalks Taking into Account Unity's Immersive Virtual Reality in an Artificial Intelligence Environment

**DOI:** 10.1155/2022/2861767

**Published:** 2022-04-10

**Authors:** Yu Hong, Yuemeng Ge

**Affiliations:** ^1^Fashion School, Zhejiang Fashion Institute of Technology, Ningbo 310058, China; ^2^Faculty of International Tourism and Management, City University of Macau, Macau 999078, China

## Abstract

In the context of the rapid development of AI area, VR technology is raising the public and researchers' attention. This study constructs a VR clothing catwalk based on the Unity 3D game engine in the AI background. This article focuses on the study of Unity 3D to construct the scenes and costumes of the clothing catwalk and then combine the immersive experience of VR to achieve the feeling of VR. Therefore, this article designs the scenes and model costumes of the VR clothing show by analyzing the VR technology in the context of the AI environment, combined with the Unity 3D game engine. It optimizes the VR clothing show based on Unity 3D game engine designed in this paper through design performance test experiment and visual positioning comparison experiment and then investigates and analyzes the optimized VR clothing show. Based on user feedback, this article completes the function of VR clothing show and compares it with the traditional online clothing show. The experimental results show that the sensory evaluation given by users is 22.02% higher than that of users of traditional online clothing shows. In the clothing catwalk based on Unity immersive VR, the user's rating for the fluency of watching is 10.99% higher than that of the traditional online clothing catwalk.

## 1. Introduction

Since the “AI” concept was promoted in 1956, the advancement and application of AI technology have achieved great success and have gradually become an important engineering technology. It is now used in automatic control, computer networks, electronic technology, and information engineering. Human beings are in the era of intelligence. Due to the application of technologies such as intelligent search engines, mechanical translation, fingerprint recognition, facial recognition, and self-discipline driving, human social life and work have become more convenient. VR technology is a simulation system which could provide virtual interaction for human beings. It uses a computer to generate a simulation environment, which is a system simulation of multisource information fusion, interactive three-dimensional dynamic visual scene, and entity behavior to make users immersed in the environment.

According to the popularization of the Internet and the development of VR technology, the VR clothing show is regarded as one of the main modes of clothing innovation. The dynamic display of clothing is an important part of the system. The design of clothing virtual catwalks based on the Unity 3D game engine can be widely used in clothing e-commerce, clothing display, and so forth, which could lead to a great impact on clothing design and marketing.

The innovation of this paper is to clarify the concept of artificial intelligence and then construct a clothing catwalks system based on the VR and AI. Designing and implementing the scenes and costumes by Unity3D game engine represent the core technology.

## 2. Related Work

The fields of neuroscience and AI have a long and intertwined history. Hassabis D. investigates the historical interaction between AI and the field of neuroscience and emphasizes the current progress of AI inspired by neural computing research in humans and other animals [1]. Hassabis D. mainly studies the interaction and combination between AI and neuroscience. That research in AI is relatively in depth, but it is insufficient in the field of VR. By studying similar inventions in the industrial, digital, and AI revolutions, Makridakis S. claims that the AI revolution is targeted; it will bring extensive changes and will also affect all aspects of society and life [2]. He has far-reaching insights and research on the AI revolution. Although his research in this area is deep, his use in the VR field is not complete. Designing a workplace can be a challenging task. It is important to ensure that the new workplace will prevent unnecessary waste of resources while also creating a safe working environment for employees. Therefore, G. Gabajová introduced a method of creating virtual workplaces using the game engine Unity 3D. Users can use VR headsets to view small details and possible shortcomings. Then it is used to visualize the strip processing to evaluate the effectiveness of the method [3]. He studied how to build a workplace by using the game engine Unity 3D to achieve VR viewing. This is very similar to the research direction of this article, but the design of the fashion show is not comprehensive enough. The success of immersive VR experiences depends on solving a large number of major challenges that span multiple disciplines. Bastug E. emphasized the importance of VR technology as a disruptive use case of 5G (and higher) that utilizes storage/memory, fog/edge computing, computer vision, AI, and other recent developments [4]. He mainly researched the impact of VR technology on 5G. If he can in-depth research on clothing catwalks, then it will be more relevant to the subject of this article. The space 4C mechanism is a two-degree-of-freedom kinematic closed chain consisting of four rigid chain links, which are simply connected in series through cylindrical (C) joints. Kihonge J. N. describes the comprehensive process of designing 4C space mechanisms in a virtual environment. VR allows users to view and interact with digital models in a more intuitive way than using traditional human-machine interfaces (HCI) [5]. Kihonge J. N.'s method of designing the 4C space mechanism in a virtual environment is very good, but it is not comprehensive enough with the clothing catwalk in this article. Mental health issues are inseparable from the environment. With the help of VR, a computer-generated interactive environment, individuals can repeatedly experience their problem situations and teach how to overcome difficulties through evidence-based psychotherapy. Freeman D. found that treatment based on VR exposure can reduce anxiety, but there are many promising research and treatment approaches [6]. His research in immersive VR focuses on mental health, and if it can involve clothing catwalks, it will be closer to the subject of this article. The 5G cellular network is considered to be a key enabler and infrastructure provider in the ICT industry by providing various services with different needs. Rongpeng tried to emphasize one of the most basic characteristics of the revolutionary technology in the 5G era, that is, the emergence of initial intelligence in almost every important aspect of the cellular network. It includes radio resource management, mobility management, and service supply management [7]. He mainly studies 5G cellular networks in the AI field, but he is not involved in the VR field. To sum up, most of the documents are AI and VR, and there are not many documents about the Unity 3D game engine designing clothing catwalks. So the focus of this article is on how to study the organic combination of VR and Unity 3D game engine.

## 3. Design Method of Clothing Catwalk System Based on Unity Immersive VR under the Background of AI

This VR system is consisted of 3 modules, and the operation flow is shown in Figure 1, which will be interpreted as follows.

### 3.1. AI Technology

AI is a branch of computer science [8]. It will create a new intelligent machine that can understand the nature of intelligence and react like human intelligence. The theory and technology of AI are transforming more mature, and technology has been applied to each area. In the future, the technological products brought by AI will become the “containers” of human intelligence [9]. It will inevitably promote the development and progress of human science and technology.

AI is a simulation of human consciousness and thinking information processing. Although AI is not human wisdom, it can react like humans, and the possibility of surpassing human wisdom will increase. AI is a very challenging science. Generally speaking, one of the main goals of AI research is to enable machines to perform complex tasks.

#### 3.1.1. Definition of Intelligence

For the realization of the concept of intelligence, the relationship between computer science and intelligence is self-evident; the most concentrated embodiment is in intelligent computing (algorithms) [10] and intelligent information processing [11]. The relationship between neuroscience and intelligence is divided into two levels, namely, the system structure level and the operating mechanism level. The most concentrated expression is in intelligent behavior and cognition. The realization of machine intelligence is based on data and algorithm, and the overall structure of neurons is the condition for human intelligence. The constant interaction and stimulation between neurons construct sensory cognition and provide an excellent model for intelligent cognition.

#### 3.1.2. AI Technology Concept

Wikipedia defines AI technology as “intelligent technology like human beings realized by ordinary computer programs.” AI technology simulates human intelligence.

AI technology is a very comprehensive subject. Due to the development and contribution of psychology, physiology, mathematics, philosophy, and other fields [5], its research and application fields have become more and more extensive. Over time, a variety of new ideas, new theories, and new technologies emerge in an endless stream. The main application field of the development of AI technology so far is the AI technology widely used in life applications. It has applications in industry, service industry, autonomous driving, medical industry, financial industry, education industry, legal industry, military, and so forth, as shown in Figure 2.

Judging from the current situation, AI can be divided into two categories: strong AI and weak AI, and we are still at the stage of weak AI. We call it “weak” because this AI itself cannot think, infer, or solve problems. That cannot be said to be intelligent in the true sense. Strong AI is the opposite. If it can cooperate with an appropriate programming language, it can theoretically perceive, think, and act independently.

There are two types of strong AI. One is human-like AI that mimics the thinking and behavior habits of humans, and the other is non-human-like AI that has its method of inference. It cannot produce and live in accordance with human thinking and action patterns. The strong AI technology is highly self-disciplined. It can act following preset instructions or decide actions according to the needs of a specific environment. It can actively handle business; that is to say, it is not set by humans in advance but can be acted on mechanically.

### 3.2. Overview of VR Technology

The definition of VR technology [12, 13] is as follows. VR technology is also regarded as spiritual technology, consisting of digital image processing, computer graphics, multimedia, graphics recognition, network, AI, sensors, and high-resolution display technology. VR is a comprehensive technology system integrating vision, hearing, touch, smell, and taste to generate three-dimensional realistic virtual environment information. The following figure clearly illustrates the five key technologies of VR technology [14] (Figure 3).

The concept of VR technology has the following meanings. First of all, from the point of view of the simulated environment, it is a computer-generated three-dimensional image that changes in real time according to a person's point of view. If it reaches the technology, in addition to the three-dimensional vision, it also includes the three-dimensional hearing, smell, touch, and other perceptions. The virtual environment is not necessarily a scene that exists in reality, but it is also a virtual world designed by the designer. From the perspective of perception, VR technology needs to theoretically simulate all human feelings, allowing users to perceive the virtual world more realistically. Finally, from the perspective of interaction, it is necessary to ensure the VR system, that is, the real-time feedback of the system, which could give people the feeling, such as the rotation of the mind and gestures; the user can naturally dialogue with the environment in the system and other users. Its application is shown in Figure 4.

In the VR system and applications, American scientists propose a triangle of VR technology including three prominent features: immersion [15], interactivity [10], and imagination [1] (Figure 5). These characteristics belong to the most important and discerning characteristics of VR technology.

#### 3.2.1. Immersion

The immersion, virtualized by computers, is used to confuse the true and false. The VR makes users feel a sense of immersion of “intentions.” Everything in the virtual world looks real and sounds real. Users will consider themselves not bystanders but participants in the virtual world. It allows the users to fully feel that they are the protagonists in the virtual environment in the process of use, thereby creating an immersive feeling. Experiencers wear interactive devices such as head-mounted smart devices and data gloves and put themselves in a virtual environment. A real three-dimensional image based on the user's physiological characteristics is generated by computers. At this point, the user will turn from an observer to participant, immersing himself in the virtual environment and becoming its member.

#### 3.2.2. Interactivity

The VR system can recognize information such as the user's language and body movements and provide real-time feedback. Users can talk with programs in the virtual world, and they can also communicate with other users as well. The information input into the system will influence the digital model of the VR system, realizing the interaction between people and programs behind the communication between people and machines. Interactivity is the embodiment of pan-AI applications in the VR field, and it is also one of the “smartest” attributes in its characteristics. The two-way nature of VR technology means “participants use natural methods to talk to the virtual environment.” The human-computer interaction function is a typical embodiment of interactivity, which represents a more harmonious and natural communication between users and the system.

#### 3.2.3. Imaginative

Not only is the VR system a digital copy of the real world but also it could be a utopia providing a rich imagination space, which is constructed from nothing. Imagination is the most interesting feature. The user can carry out a series of thinking processes such as association and reasoning based on the information obtained from interaction logs and imagine the future of the system movement as the system changes. In this process, the users can produce rich imagination and take an interesting journey of imagination. The VR system also broadens the scope of human cognition and stimulates human imagination.

### 3.3. Unity 3D

Unity [2, 7] is a 3D-based, cross-platform engine. The biggest advantage of Unity 3D is that it allows artists and coders to coordinate their work in a unified environment. It is a user-friendly, convenient, and fast development tool. The object engine in the Unity engine brings realistic physical effects in the real world to the game world. It can add a collider component to the objects in the scene and use it to detect whether there is an interaction between two objects in real time. Also, Unity 3D provides a simple and easy-to-use development and editing interface and highly aggregated script editing. It can recognize model formats exported by a variety of 3D modeling software and can recognize model textures, animations, and bone bindings of characters. For example, Maya, 3D Studio Max, Cheetah, Cinema4D, Blender, Carrara, Lightwave, XSI, and Modo may be more compatible later, which greatly reduces the barriers to use for developers.

#### 3.3.1. Unity 3D Features

As the most popular open-source engine, Unity 3D has the following characteristics:

1. It supports visual editing and hierarchical integrated development environment and can have a rich element checker and real-time preview of works.
2. Diversified export platforms. Unity can directly export the produced content as .exe files under the Windows platform and .dmg files under the OSX platform. In addition, through the Unity Web Player plug-in, resources can also be directly exported to the browser for direct use.
3. Automatically import resources. In Unity, it can directly import design models or scripts into the Unity editor by dragging and dropping. The external changes of resources will also be updated in real time in the project. Unity 3D supports most of the current mainstream 3D modeling formats, such as 3DMax and SketchUp, and other software design drafts can be seamlessly docked, giving developers greater convenience for the use of third-party models.
4. Unity uses the current popular and compatible graphics library, for example, Microsoft Direct and OpenGL, and built-in support for Nvidia's PhysX physics engine [16].
5. The development of game scripts is based on the cross-platform open-source version Mono of Microsoft .NET Framework. With Unity's built-in API support, developers can execute scripts by writing JavaScript and C#.
6. Unity uses widely supported video and audio formats and can compress some media files based on the purpose of game development. In addition, Unity also has many built-in resources and includes a powerful official application store. It supports multiperson network connection function, provided by a third-party package; there are many options such as RakNet, Photon, and SmartFoxServer.

#### 3.3.2. The Core Module of the Unity 3D Engine

The Unity 3D engine mainly has 4 core modules, and the main functions of each module are as follows:

1. Object module: Various elements, scenes, and buttons in the stage are all stage objects. The object is the most basic unit of stage production and can be assigned to the corresponding script code.
2. Event processing module: By changing various attributes of the stage object, the state of each element of the stage is changed. The event processing module is used to change the attributes of the level object.
3. Camera module: The concept of camera comes from 3D stage design. The content displayed by the user on the device will change with the content of the camera. The position and angle of the camera are controlled by scripts, and the user can confirm changes to the stage interface, scene, and role. The switching of stage scenes is usually realized by controlling the switches of various cameras.
4. Rendering module: The rendering module performs real-time calculation of all effects such as models, animations, lighting, and special effects and displays them on the screen. The presentation module is the most complex of all modules, and its ability directly determines the final output quality of the stage.

#### 3.3.3. Features of Clothing Catwalks Based on Unity 3D Design

1. The system structure is reasonable, concise, and clear, which can meet the target needs of the subject.
2. High system reliability. For the user to restart the device, it can continue to rerun the system according to the default method for experience.

### 3.4. Immersive Display Module Design

The nonconvergent binocular imaging model [17, 18] is a three-dimensional display model constructed based on the principle that humans use binocular parallax to generate stereo vision, as shown in Figure 6.

We have that *O*, *O*′ simulate the left and right focus positions of the human eye, the distance is *D*, the human line of sight is parallel to the *c*-axis, and the left and right images seen by the human eye are perpendicular to the *c*-axis and parallel to the *ab* plane. The focal length of the simulated human eye is *f*. Assuming that there is a three-dimensional coordinate point *Q* (*a*, *b*, *c*) in the distance, the points presented on the left and right image planes are *Qd* and *Qr*. Among them, the parallax *l* of the point *Q* formed by *Qd* and *Qr* is |*Qr*−*Qd*|; then

(1) $$\begin{array}{c} \left(a,b,c\right)=\frac{D}{l\left(a^{\prime },b^{\prime },f\right)}. \end{array}$$

Point (*x*′, *y*′) is the coordinate of point *Pl* mapped by point *P* on the left image plane, where the relationship between *d* and *z* is

(2) $$\begin{array}{c} l=\frac{Df}{c}. \end{array}$$

As shown in Figure 7, the projection plane is parallel to the *xy* plane and is at a distance *d* from the origin on the *z*-axis.

The range of independent projection plane coordinates is summed. Then, the parametric formulas of the projection lines of points −1 ≤ *a* ≤ 1, −1 ≤ *b* ≤ 1, and DCoQ can be obtained:

(3) $$\begin{array}{c} c=c_{0}+t\left(0-c_{0}\right),\\ b=b_{0}+t\left(0-b_{0}\right),\\ a=a_{0}+t\left(\frac{q}{2}-a_{0}\right). \end{array}$$

Substituting the view plane *z* = *l* into the formula yields

(4) $$\begin{array}{c} t=\frac{c_{0}-l}{c_{0}}. \end{array}$$

The projection point coordinate (*a*_*d*_, *b*_*d*_) of DCoQ on the projection plane is

(5) $$\begin{array}{c} b_{d}=\frac{lb_{0}}{c_{0}},\\ a_{d}=\frac{la_{0}}{c_{0}}-\frac{ql}{2c_{0}}+\frac{q}{2}. \end{array}$$

In the same way, the coordinate (*a*_*r*_, *b*_*r*_) of the projection point generated by the projection line of point *Q*_0_(*a*_0_, *b*_0_, *c*_0_) and RZoQ in the projection plane is

(6) $$\begin{array}{c} b_{r}=\frac{lb_{0}}{c_{0}},\\ a_{r}=\frac{la_{0}}{c_{0}}-\frac{ql}{2c_{0}}-\frac{q}{2}. \end{array}$$

Due to *b*_*d*_=*b*_*r*_, the horizontal parallax between the left and right imaging viewpoints is

(7) $$\begin{array}{c} H=a_{d}-a_{r}=-\frac{ql}{c_{0}}+q. \end{array}$$

On the left side of the calculation point *Q*_0_(*a*_0_, *b*_0_, *c*_0_), the imaging position is shifted along *a* by −q/2, so that

(8) $$\begin{array}{c} Q_{0\text{left}}=\left(a_{0}-\frac{q}{2},b_{0},c_{0}\right),\\ Q_{0\text{right}}=\left(a_{0}+\frac{q}{2},b_{0},c_{0}\right). \end{array}$$

The parametric formula of the projection line from *A* to the projection center is

(9) $$\begin{array}{c} c=c_{0}+t\left(0-c_{0}\right),\\ b=b_{0}+t\left(0-b_{0}\right),\\ a=a_{0}+\frac{q}{2}+t\left[0-\left(\frac{q}{2}+a_{0}\right)\right]. \end{array}$$

At the viewing plane *z* = *l*,

(10) $$\begin{array}{c} t=\frac{\left(c_{0}-l\right)}{c_{0}}. \end{array}$$

Then,

(11) $$\begin{array}{c} b_{r}=\frac{lb_{0}}{c_{0}},\\ a_{r}=\frac{la_{0}}{c_{0}}-\frac{ql}{2c_{0}}. \end{array}$$

In the same way, for *Q*_0left_,

(12) $$\begin{array}{c} b_{d}=\frac{lb_{0}}{c_{0}},\\ a_{d}=\frac{la_{0}}{c_{0}}-\frac{ql}{2c_{0}}. \end{array}$$

The horizontal disparity is expressed as a difference:

(13) $$\begin{array}{c} \left(a_{d}-a_{r}\right)=\frac{-ql}{c_{0}}. \end{array}$$

Here, since *c*_0_ is always greater than zero, we get that the value of disparity is always negative, so the image will be presented in front of the projection surface.

## 4. Test Experiment of Clothing Catwalk System Based on Unity Immersive VR under the Background of AI

### 4.1. Performance Test Experiment

Through the analysis of the server log, the client's request is calculated, and all these requests (URL) are used as the input of siege to test the load capacity of a single terrain server. 25 tests were performed, and the number of simultaneous executions was gradually increased from 5 to 500 and the step size was increased from 5 to 50. Each exam lasted 20 seconds. These four indicators change with time in each test. To test accuracy, the average value of the indicators in the test is used for comparison. The server memory is 16G, and the memory usage in the test is not high. Therefore, in this experiment and testing process, there is no need to pay attention to the memory occupancy rate. The test results are shown in Figure 8.

As shown in Figure 8, if the number of simultaneous executions increases from 5, the throughput rate of the server will also increase rapidly, but the increase rate will slowly decrease. In the process of increasing the number of simultaneous executions from 50 to 500, the throughput rate is relatively stable at 6300 reqs/s, the data throughput rate is relatively stable above 100 MB/s, and the CPU occupancy rate changes within a small range, about 55%.

When the number of simultaneous executions is 300, the data throughput rate reaches the maximum value of 109.21 MB/sec. Since the tested network environment was a 1 Gbps local area network, it basically reached the theoretical maximum value of data transmission. Therefore, in this case, the performance of the CPU is not a bottleneck but is limited by the network bandwidth, and the throughput is further increased. If the network bandwidth allows, it needs to increase the number of requests processed by 1 second.

After the concurrent number exceeds 400, both the throughput rate and the data throughput rate have a slow downward trend. This shows that the server's ability to handle concurrent connections is still limited. Excessive concurrency will bring additional burdens to the server and affect its processing capabilities. The throughput test data of the two results are shown in Tables 1 and 2.

Test results show that the size returned by URL2 is about 28 KB, which is much larger than URL1. Therefore, it can fill up the entire network bandwidth, the data throughput rate can reach about 100 MB/s, and it can basically remain stable when the number of concurrent connections is from 10 to 2000.

On the other hand, the returned result size is small in Table 1, and its bottleneck is in other aspects, such as CPU. In the process of testing URL1, the CPU occupancy rate was relatively high, basically maintained at about 90%. Other bottlenecks may be the operating speed of the database (mainly cache Redis) [19]. Nevertheless, the server can still handle more than 14,000 requests per second in the best case, indicating that the system performance is still good.

By tracking the user's access behavior, we have calculated a user's call to the server API in 10 minutes, and the statistical results are shown in Table 3 and in Table 4.

In summary, for the LBS data changes frequently, the cache and the database are prone to data inconsistencies, so the implementation of the cache system is difficult. Without using the cache, the pressure of LBS service will transfer to be on the database, while it also has a higher requirement on the CPU computing power. Therefore, its throughput rate is lower than that of services with simple logic such as terrain services. To improve the performance of the LBS service, it is necessary to use the cache, which can greatly reduce the pressure on the database, while reducing the response time and returning the results to the client faster. On the other hand, it is necessary to optimize the system and reduce string operations, which could reduce CPU usage and improve the server's ability to process requests.

### 4.2. Visual Positioning Contrast Experiment

Using the method proposed in this article to carry out the experiment, in the process of walking along the positive direction of the *x*-axis, when walking to a fixed position, it suddenly accelerates back and forth. After many rounds, for the same segment of the walking process, respectively use the visual positioning method based on the logo and the method in this paper to conduct experiments. For different walking distances, the single frame refresh time was compared, and the experimental results obtained are shown in Table 5.

Since the maximum acquisition speed of the camera used in the experiment is 30 frames per second, the speed of the visual tracking algorithm is also limited by the performance of the camera to a certain extent. Aiming at the experimental scene in this article, 1000 frames of images are recognized, and the tracking results are shown in Table 6.

The main purpose of this experiment is to verify whether the improved tracking algorithm can choose different threshold segmentation methods according to different lighting environments and achieve better experimental results. The experimental scene is shown in Figure 9, which ensures that the camera can only shoot a complete mark at any position. When the user moves along the *x*-axis direction, it will experience two uneven illumination situations: observe the positioning results and compare them with the visual positioning method based on signs.

When the visual tracking algorithm based on fixed threshold segmentation is used, it will fail to locate near the light source. Figure 9 shows that there are indeed three pieces of data which fail to locate. However, the method in this paper is robust to the ambient lighting. When the camera collects the image close to the light source, the local adaptive threshold segmentation method will be activated, which can ensure the accuracy and continuity of the positioning.

## 5. Investigation and Analysis of Clothing Catwalk System Based on Unity Immersive VR in AI Environment

### 5.1. Investigation and Analysis of System Design

Comprehensive, rigorous, and standardized tests have been carried out in the user's field environment in terms of function, performance, environment, reliability, and user interface. It designs system analysis and testing programs, as well as fluency and immersion-related test surveys, and determines the expected requirements of the software in terms of functional use cases and nonfunctional goals of the system based on the displayed results. It meets the relevant design requirements. The results of the survey are shown in Figure 10.

Figure 10 reveals that, in the aesthetic evaluation of the interface, 25 people reckon that the aesthetics of the system UI are remarkable, and 13 people consider it is very good; only 2 people think it is just good. This shows that fine UI will achieve popularity among the public. In the system simulation evaluation, 21 people reckon it is excellent, 13 people regard it is excellent, and 6 people think it is good. This shows that the system simulation is not bad. In the evaluation of system immersion, 18 people reckon it is excellent, 18 people consider it is very good, and only 4 people think it is good. This shows that the system immersion is very good. In the level of system flow, 12 people think it is very good, and the rest think it is relatively good, which shows that the smoothness of the system is very popular with the public.

### 5.2. Comparative Analysis between the Design of Unity-Based Immersive VR Clothing Catwalks and Traditional Online Clothing Catwalks under the Background of AI

Combining the data obtained from the performance experiment to optimize the clothing catwalk designed in this paper, in order to verify the improvement of traditional online clothing catwalks, this study compares the optimized clothing catwalks based on VR and traditional online clothing catwalks through user sensory and fluency scores. We collect 100 evaluations and select 10 to compare the scores of the two clothing selections randomly. The experimental results are shown in Figure 11.

As shown in Figure 11, in the clothing show based on VR system supported by AI, the sensory evaluation given by users is 93.15 points, while that of the traditional online clothing catwalks is only 76.34 points. It can be seen that the costume show based on VR system has a 22.02% improvement in user senses compared to the traditional online costume show. In the clothing show based on VR system, the user gave a score of 90.58 points for viewing fluency, while the traditional online clothing show user gave only 81.61 points for watching fluency. It can be seen that the clothing show based on VR system has a 10.99% improvement in viewing fluency compared with the traditional online clothing show. The experimental results show that the costume show based on VR system has greatly improved the sense and fluency of users compared with the traditional online clothing show.

## 6. Limitation and Conclusions

This article mainly studies the design of a VR clothing catwalk in the context of the AI environment combined with the Unity 3D game engine, so this paper focuses on the design of a VR clothing catwalk based on the Unity 3D game engine. By understanding the characteristics of VR under the background of AI, this article deeply studies the immersive experience of VR technology and designs a VR clothing show based on Unity 3D game engine. Through the scene rendering of the Unity 3D engine, the scene and clothing design can be more realistic, and the user's senses are becoming more and more realistic. In order to verify the performance of the VR clothing show based on the Unity 3D game engine designed in this article, this paper designs a performance test experiment and a visual positioning comparison experiment to optimize the VR clothing show based on the Unity 3D game engine. Then, through the investigation of the analysis system design, a comparative experiment with traditional online clothing catwalks was designed. Experimental results show that the design of VR clothing catwalks based on Unity 3D game engine has a stronger user sensory experience and smoother screen design than traditional online clothing catwalks.

The major limitation of the present study is that the dimension designed for the VR clothing show is relatively single. This article only studies the visual modality as VR, but, in the metaverse stage, multimodal access will greatly enhance the immersive feeling of VR show. So, future research should be undertaken to explore the brain-computer interaction and touch simulation to construct a more immersive VR interaction situation.

## Figures and Tables

**Figure 1:** VR system modules.

**Figure 2:** Application of AI technology.

**Figure 3:** VR key technologies.

**Figure 4:** Application of VR technology.

**Figure 5:** The triangle of VR technology.

**Figure 6:** Binocular vision model.

**Figure 7:** Schematic diagram of dual center projection.

**Figure 8:** Experimental test results.

**Figure 9:** Comparison of positioning results between the method in this paper and the visual positioning method based on signs in a changing lighting environment.

**Figure 10:** System experience survey results.

**Figure 11:** Comparison results of clothing catwalks based on Unity immersive VR and traditional online clothing catwalks.

**Table 1:** URL1 test results.

	URL1, 1756 bytes	
Concurrency	Throughput rate (reqs/s)	Data throughput rate (MB/s)
10	10514.94	19.42
100	13548.44	24.64
1000	14034.06	25.66
2000	12394.67	24.33

**Table 2:** URL2 test results.

	URL2, 28585 bytes	
Concurrency	Throughput rate (reqs/s)	Data throughput rate (MB/s)
10	3649.21	103.11
100	4089.16	114.66
1000	4064.81	11.65
2000	4083.46	114.32

**Table 3:** Statistics of API calls.

API	Frequency	Instruction
/Account/login	1	User login
/Comments/friends_timeline	2	Get good comment timeline
/Comments/poi_timeline	1	Get POI comment timeline
/Pois/list	24	Get a list of POIs in a certain area

**Table 4:** LBS service test data.

Concurrency	Throughput rate (reqs/s)	Data throughput rate (MB/s)	CPU usage (%)		Average response time (s)
			#1 (%)	#2 (%)	
10	1324.61	4.81	79.36	14.64	0.01
20	1945.18	7.10	93.41	32.49	0.01
30	1994.67	7.16	93.84	26.54	0.01
40	1976.45	7.00	94.41	22.64	0.02

**Table 5:** Comparison of single frame time consumption between the positioning method in this paper and the visual positioning method based on the logo for different walking distances.

Walking distance/m	Representation-based visual positioning method	Method of this article
2.5	8.331	8.874
5	8.416	9.154
10	10.131	10.644

**Table 6:** The performance comparison of the method in this paper, the fixed threshold, and the adaptive threshold tracking method.

method	Recognition rate (%)	Single frame time (ms)
Fixed threshold visual tracking	56	51
Adaptive visual tracking	98.8	126
Method of this article	97.4	73

## Data Availability

The data used to support the findings of this study are available from the corresponding author upon request.
